The article "Regulation of the Keap1-Nrf2 Signaling Axis by Glycyrrhetinic Acid Promoted Oxidative Stress-Induced H9C2 Cell Apoptosis" was published in 2022. Journal: Evid Based Complement Alternat Med.

# Regulation of the Keap1-Nrf2 Signaling Axis by Glycyrrhetinic Acid Promoted Oxidative Stress-Induced H_9_C_2_ Cell Apoptosis

**DOI:** 10.1155/2022/2875558

**Published:** 2022-08-27

**Authors:** Zhangyu Jiang, Yanqing Wang, Xiuli Xi, Weibin Cai, Changhui Liu, Ran Ye, Liu Yang, Song Zhang, Rong Zhang, Qin Xu, Lei Yang

**Affiliations:** ^1^Guangzhou University of Chinese Medicine, Guangzhou, China; ^2^Research Center of Integrative Medicine, School of Basic Medical Sciences, Guangzhou University of Chinese Medicine, Guangzhou, China; ^3^School of Pharmaceutical Sciences, Guangzhou University of Chinese Medicine, Guangzhou, China

## Abstract

Excessive reactive oxygen species (ROS) could interfere with the physiological capacities of H_9_C_2_ cells and cause cardiomyocyte apoptosis. Glycyrrhetinic acid (GA), one of the main medicinal component of *Glycyrrhetinic Radix* et *Rhizoma*, shows toxic and adverse side effects in the clinic setting. In particular, some studies have reported that GA exerts toxic effects on H_9_C_2_ cells. The purpose of this study is to assess the effect of GA-induced oxidative stress on cultured H_9_C_2_ cells and reveal the relevant signaling pathways. LDH assay was used to assess cell damage. Apoptosis was detected using Hoechst 33242 and a propidium iodide (PI) assay. An Annexin V-fluorescein isothiocyanate/PI double-staining assay was utilized to investigate GA-induced apoptosis in H_9_C_2_ cells. The expression level of specific genes/proteins was evaluated by RT-qPCR and Western blotting. Flow cytometry and DCFH-DA fluorescent testing were used to determine the ROS levels of H_9_C_2_ cells. The potential mechanism of GA-induced cardiomyocyte injury was also investigated. GA treatment increased ROS generation and mitochondrial membrane depolarization and triggered caspase-3/9 activation and apoptosis. GA treatment also caused the nuclear translocation of NF-E2-related factor 2 after its dissociation from Keap1. This change was accompanied by a dose-dependent decline in the expression of the downstream target gene heme oxygenase-1. The findings demonstrated that GA could regulate the Keap1-Nrf2 signaling axis and induce oxidative stress to promote the apoptosis of H_9_C_2_ cells.

## 1. Introduction

As an organ with a high energy demand, the heart is especially abundant in mitochondria and organelles that play a vital part in energy metabolism and other cellular activities, such as cell proliferation, reactive oxygen species (ROS) degradation, and cell apoptosis [1]. Over the last 60 years, 462 drugs worldwide have been pulled from the market because of their toxic effects. Death and liver, heart, and nervous system toxicity are among the main reasons behind the withdrawal of drugs [2]. Cardiac safety evaluation is a major concern in the clinical research of new drugs. A total of 14 drugs that could cause torsade de pointes ventricular tachycardia have been withdrawn from the global market [3]. Drug-induced cardiotoxicity is a key issue, and cardiotoxicity events may occur even after a drug is marketed [4]. Therefore, the cardiotoxicity of drugs is a cause for great concern among clinicians, medical researchers, and pharmaceutical companies.

The article "Regulation of the Keap1-Nrf2 Signaling Axis by Glycyrrhetinic Acid Promoted Oxidative Stress-Induced H9C2 Cell Apoptosis" was published in 2022. Journal: Evid Based Complement Alternat Med.

Multiple studies have linked drug-induced cardiotoxicity to excesses in ROS generation, which implies that oxidative stress is a motivating factor in cardiomyocyte apoptosis, leading to heart failure [5]. And the current accepted view on the production of oxidative stress is that excessive free radicals are produced by the body after injury. When a large number of highly active molecules are released into the bloodstream, the body's antioxidant capacity is reduced, and excessive oxidative substances accumulated in the body cannot be eliminated. This process leads to a dynamic imbalance between the oxidation and antioxidant systems, resulting in tissue damage. And the most important endogenous antioxidant signaling pathway in the body is the Keap1-Nrf2 signaling pathway [6]. The transcription factor Nrf2 as well as its cytoplasmic adaptor protein Keap1 have been identified as key mediators of the cellular antioxidant reaction in recent investigations. When the Keap1-Nrf2 signaling axis is attacked by ROS and nucleophiles, it regulates antioxidant enzyme proteins [7]. The accumulation of significant amounts of active oxygen produced by oxidative stress in the body induces all kinds of cardiovascular illnesses, including heart failure and atherosclerosis.

The mitochondria are the primary energy source of cells, which play an important role in cell death. As an abundant component of cardiomyocytes, mitochondria govern the cell cycle, metabolism, and signal transduction. Arrhythmia, heart failure, and other cardiovascular disorders are affected by cardiomyocyte apoptosis [8]. The mechanism of the cardiotoxicity of many drugs, such as cisplatin and Adriamycin, is related to mitochondrial apoptosis. In the myocardial injury caused by Adriamycin, the expression of Bax, caspase-3, and cleaved PARP increases whereas the expression of Bcl-2 decreases, thus demonstrating that the cardiotoxicity of Adriamycin is closely related to apoptosis [9, 10]. And apoptosis is a controlled adenosine triphosphate-dependent process in which aggregated caspase is activated as a consequence of the lack of mitochondrial membrane potential (MMP; i.e., the innate route) or activation of the tumor necrosis factor receptor (i.e., the extrinsic route) [11, 12]. Numerous studies have shown that mitochondria are efficient energy sources and that mitochondrial malfunction could be linked to the etiology of cardiotoxicity [13, 14]. Various lines of evidence suggest that mitochondrial-related toxicity, whether direct or indirect, is a matter of normal mechanism of direct drug-induced cardiotoxicity. Interference with the mitochondrial respiratory chain or obstruction of critical mitochondrial enzymes may cause mitochondrial toxicity, facilitate the generation of ROS and calcium excess, and induce the opening of mitochondrial permeability transition pores. These processes eventually induce apoptosis and/or cell necrosis.

The article "Regulation of the Keap1-Nrf2 Signaling Axis by Glycyrrhetinic Acid Promoted Oxidative Stress-Induced H9C2 Cell Apoptosis" was published in 2022. Journal: Evid Based Complement Alternat Med.

*Glycyrrhetinic Radix* et *Rhizoma* refers to the dry rhizomes of *Glycyrrhiza glabra L.*, *Glycyrrhiza uralensis Fisch.*, and *Glycyrrhiza inflata Batalin.* [15], whose main active ingredients include saponins, polysaccharides, and flavonoids [16–18]. And GA is the main component of saponins and has anti-inflammatory, antibacterial, and anticancer effects [19, 20]. What's more, GA is one of the main hydrolyzed active components of *Glycyrrhetinic Radix* et *Rhizoma* in the body [21, 22].

Long-term consumption of GA can cause increases in blood pressure, retention of water and sodium, excretion of potassium ions, and slight reductions in the sodium/potassium ratio in urine. And this effect is similar to that of aldosterone [23, 24]. The toxic and side effects of GA limit its wider application in the market and clinical setting. However, the toxic effect of GA on H_9_C_2_ cardiomyocytes has not been well documented. In this study, we examined the effects of GA on H_9_C_2_ cells *in vitro*. And we also investigated whether oxidative stress-induced myocardial apoptosis is modulated by changes in the Keap1-Nrf2 signaling pathway following GA treatment. The results of this work could bring about a greater comprehending of the molecular mechanisms of GA within the therapeutic limit for cardiotoxicity.

## 2. Materials and Methods

### 2.1. Antibodies and Reagents

GA (≥98% purity; molecular formula, C_30_H_16_O_4_; molecular weight, 470.69; CAS No. 471-53-4) was purchased from Chengdu Pufei De Biotech Co., Ltd., China. GA was dried under reduced pressure at 60°C for 2 hours before use, dissolved in DMSO, and used immediately after preparation. Cell Counting Kit-8 (CCK-8) assay kits were obtained from Dojindo (Japan). The Annexin V-fluorescein isothiocyanate (FITC)/propidium iodide (PI) apoptosis detection kits were obtained from BestBio Institute of Biotechnology (Shanghai, China). Antibodies against Keap1 (AF5266, 1 : 1000 dissolution), Nrf2 (AF0639, 1 : 1000 dissolution), HO-1 (AF5393, 1 : 1000 dissolution), Bax (AF0120, 1 : 2000 dissolution), Bcl-2 (AF6139, 1 : 1000 dissolution), PCNA (AF0239, 1 : 5000 dissolution), *β*-actin (TA0022, 1 : 3000 dissolution), and GAPDH (AF7021, 1 : 5000 dissolution) were obtained from Affinity Biosciences (OH, USA). Cell Signaling Technology, Inc. (Boston, MA, USA) provided the primary antibodies against cleaved Caspase-3 (9664, 1 : 1000 dissolution) and PARP (9532s, 1 : 1000 dissolution). Abcam (Cambridge, UK) provided the antibodies against caspase-9 (ab184186, 1 : 2000 dissolution).

The article "Regulation of the Keap1-Nrf2 Signaling Axis by Glycyrrhetinic Acid Promoted Oxidative Stress-Induced H9C2 Cell Apoptosis" was published in 2022. Journal: Evid Based Complement Alternat Med.

### 2.2. Cell Culture

The cardiomyoblast H_9_C_2_ cells were taken from the Cell Bank of the Chinese Academy of Sciences (Shanghai, China). Neonatal rat ventricular myocytes (NRVMs) were primarily isolated from neonatal (1-2 d) Sprague–Dawley rat hearts that is frequently used to assess cardiotoxicity *in vitro* [25]. These cells were cultivated in 25 cm^2^ tissue culture flasks in a humidified atmosphere of 5% CO_2_ at 37°C in Dulbecco's modified Eagle's medium (DMEM). The cell cultures were supplemented with fresh medium every 2-3 d. When cells reached 80–90% confluence, the cell culture medium was removed and the cells washed with prewarmed phosphate-buffered saline (PBS). Then cultures were passaged by trypsinization (0.25% trypsin/1 mM EDTA solution) and subcultured over a maximum of 10 passages.

### 2.3. Cell Viability Assay

To assess the cell viability and proliferation, the CCK-8 assay was utilized. In brief, H_9_C_2_ cells were gathered and planted at a density of 5 × 10^4^ cells/well in 96-well plates. After the various treatments, cells were incubated with 10 *μ*L CCK-8 solution for 1 h following the manufacturer's specification. The data was evaluated by detecting the optical density (OD) at 450 nm using a microplate reader (PerkinElmer EnSpire, USA).

### 2.4. LDH Activity Assay

GA was given to H_9_C_2_ cells for 24 or 48 hours. A kit was used to identify LDH activity, which was done according to the manufacturer's instructions. 1 h before the scheduled detection time point, the cell culture plate was removed from the cell culture box and LDH release reagent was added, repeated blowing and mixed several times, and then the cell culture plate continued to incubate in the cell culture box. After reaching the preset time, the liquid in the 96-well plate was collected into a 0.5 mL EP tube and centrifuged at 400*g* for 5 min. 120 *μ*L supernatant of each EP tube was added to the corresponding well of a new 96-well plate, and samples were determined immediately. 60 *μ*L of LDH detection working solution was added to each sample, and after mixing, each sample was incubated at room temperature (about 25°C) for 30 minutes in the dark, and slowly shaken on a horizontal shaker. Finally, the absorbance was measured at 490 nm and calculated.

The article "Regulation of the Keap1-Nrf2 Signaling Axis by Glycyrrhetinic Acid Promoted Oxidative Stress-Induced H9C2 Cell Apoptosis" was published in 2022. Journal: Evid Based Complement Alternat Med.

### 2.5. ROS Assay

We employed the DCFH-DA as a tag to examine the generation of intracellular ROS, as per the manufacturer's recommendations. Put simply, H_9_C_2_ cells were grown for 48 h on glass cover slips in six-well plates. Following GA treatment, the H_9_C_2_ cells were washed thrice with PBS and then incubated in serum-free medium with 10 *μ*M DCFH-DA for 40 min at 37°C in the darkness. Moreover, a fluorescent microscope (Leica, Germany) was used to examine the cells. The H_9_C_2_ cells were collected, resuspended in flushing solution at a concentration of around 2 × 10^5^ cells/mL, incubated with DCFH-DA, and then examined using a flow cytometer with a 500 nm excitation filter and a 530 nm emission filter.

### 2.6. Hoechst 33242 and PI Assay

H_9_C_2_ cells were sown on a coverslip, treated with GA, and fixed with 1% Hoechst 33342 and 1% PI solution at 4°C for 10 min in the dark. The slides were washed thrice with cold PBS and then incubated with 4 *μ*L of antifluorescence quenching reagent. Photographs were obtained with a fluorescence microscope (Leica) in the last step.

### 2.7. Flow Cytometry

H_9_C_2_ cells were harvested using 0.25% trypsin at 37°C, treated with GA for 24 h, and then washed thrice with cold PBS (1000 rpm, 3 min). Approximately 1 × 10^6^ cells were resuspended in 500 *μ*L of fresh binding buffer and treated with 5 mL of Annexin V-FITC and 5 mL of PI solution for 15 min at ∼25°C. In the last step the flow cytometry was used to examine the FL1 (FITC) and FL3 (PI) laser lines of the treated samples.

### 2.8. Mitochondrial Membrane Potential (MMP) Analysis

Changes in the MMP of the H_9_C_2_ cells after GA treatment were assessed by JC-1 staining. Briefly, H_9_C_2_ cells were treated with GA (15–45 *μ*M) for 24 h, rinsed thrice with cold PBS, and then incubated with JC-1 solution for 20 min in a conventional cell incubator. The H_9_C_2_ cells were then washed twice with JC-1 staining buffer (1×) for 3 min each time. A fluorescent microscope (Leica) was used to photograph H_9_C_2_ cells stained with JC-1 solution.

### 2.9. Western Blotting

Entire cell extracts (30 *μ*g) were treated with 0.45 *μ*M GA, separated using SDS at 80 V for 1.5–2 h at ∼25°C, then electro-transferred onto PVDF membranes at 300 mA for 90 min at 4°C. The PVDF membranes were washed thrice with TBST (1×) for 5 min each time, blocked with 5% nonfat dry milk in TBST (1×) for 2 h at approximately 25°C, rinsed with TBST (1×), incubated with the main antibodies for 12 h at ∼4°C, and then washed thrice with TBST (1×), incubated with HRP-linked anti-IgG for 1 h at approximately 25°C, and next washed thrice with TBST (1×). GAPDH, *β*-actin, and PCNA served as controls. The chemiluminescent bands of the membranes were finally examined using ChemiDoc XRS + (Bio-Rad, USA) software, and the blots were evaluated by Image J.

The article "Regulation of the Keap1-Nrf2 Signaling Axis by Glycyrrhetinic Acid Promoted Oxidative Stress-Induced H9C2 Cell Apoptosis" was published in 2022. Journal: Evid Based Complement Alternat Med.

### 2.10. Quantitative Real-Time PCR

After treating the H_9_C_2_ cells with GA, total RNAs were extracted using TriZol (Takara Biotechnology, Japan). After confirming the concentration of each RNA group, PrimeScript™ RT Master Mix (Takara) was used to reverse-transcribe 500 ng of total RNA samples into cDNA. Afterward, each test was subjected to real-time PCR according to the manufacturer's instructions of Keap1, Nrf2, and GAPDH using the double-stranded DNA dye SYBR Premix Ex Taq™ II kit (Takara). The PCR program was as described in the following: starting denaturation of 35 s at 95°C, followed by 40 cycles of 30 s at 60°C. GAPDH (Shenggong Biotech, China) served as the control. The primers used were as follows:

  Keap1 forward, 5′-CATCGGCATCGCCAACTTC-3′;
  Keap1 reverse, 5′-GCTGGCAGTGTGACAGGTTGA-3′;
  Nrf2 forward, 5′-TTGGCAGAGACATTCCCATTTGTA-3′;
  Nrf2 reverse, 5′-GAGCTATCGAGTGACTGAGCCTGA-3′;
  GAPDH forward, 5′-GGCACAGTCAAGGCTGAGAATG-3′;
  GAPDH reverse, 5′-ATGGTGGTGAAGACGCCAGTA-3′;

The data were evaluated using the 2^−∆∆Ct^ method after RT-qPCR was done using triplet rehash PCR.

### 2.11. Statistics

All data are presented as the mean ± SD and analyzed by one-way ANOVA followed by the LSD test (*n* = 3). Statistical significance was defined as a *P* value of <0.05. SPSS 13.0 software was used to conduct all statistical analyses.

## 3. Results

### 3.1. GA-Induced H_9_C_2_ Cell Damage

Figure 1(a) is the structure of GA. In the first place, we examined the effect of GA on the viability and proliferation of H_9_C_2_ cells. GA suppressed the proliferation of H_9_C_2_ cells in a time- and dose-dependent manner, as shown in Figure 1(b). CCK-8 assay revealed a decrease in cell viability to approximately 74% after treatment with 45 *μ*M GA for 48 h. LDH leakage, a marker of cell damage caused by plasma membrane breakdown, was significantly increased after GA treatment (Figures 1(c) and (d)), showing that the control group has tightly packed membranes and a regular cell shape. By contrast, cells that had been exposed to GA had poorly packed membranes and displayed signs of shrinkage.

### 3.2. The Mitochondrial Pathway Played a Critical Role in the Apoptosis Induced by GA

We sought to define if the cytotoxic activity of GA is associated with apoptosis. And flow cytometry, Hoechst 33242, and PI assays were used to detect apoptosis in H_9_C_2_ cells. The results indicated that H_9_C_2_ cells treated with GA have higher apoptotic rates than control cells and that cell death occurs in a concentration-dependent way (*P* < 0.05). When the H_9_C_2_ cells were treated with 45 *μ*M GA, the population of apoptotic cells increased by 12.13% (*P* < 0.05; Figures 2(b) and 2(c)). And Hoechst 33242 and PI assays revealed brighter nucleus staining, nuclear chromatin condensation, and karyorrhexis, thereby indicating that the GA-treated groups have higher cell apoptosis rates than the control groups. As the GA concentration increased, the blue fluorescence in the cells became brighter. This result indicates that cardiomyocytes undergo apoptosis after GA administration and that the effects of GA are dose-dependent (Figure 2(a)).

The article "Regulation of the Keap1-Nrf2 Signaling Axis by Glycyrrhetinic Acid Promoted Oxidative Stress-Induced H9C2 Cell Apoptosis" was published in 2022. Journal: Evid Based Complement Alternat Med.

After 24 h of treatment with 15, 30, and 45 *μ*M GA, the levels of PARP, caspase-3, and caspase-9 were measured to define the apoptotic response of cells to GA treatment. Compared with the control, the GA-treated groups showed dose-dependent improvements in the cleavage of caspase-3 and caspase-9 (*P* < 0.05). And cleavage of PARP occurred in a similar manner (*P* < 0.05; Figures 3(a) and 3(b)). These findings confirm that GA promotes cell apoptosis in H_9_C_2_ cells in a dose-dependent way.

A reduction in MMP could trigger a cascade of apoptotic procedures. MMP was measured by JC-1 staining to determine whether GA-induced apoptosis is linked to the MMP pathway in H_9_C_2_ cells. Regular mitochondria displayed red fluorescence following JC-1 labeling, as seen in Figure 4(a). And H_9_C_2_ cells treated with GA initially revealed green fluorescence, which indicates a reduction in MMP, followed by a drop in red/green fluorescence ratio, which is associated with apoptosis. H_9_C_2_ cells treated with 15, 30, and 45 *μ*M GA demonstrated increased MMP loss as compared to the control group. The deficiency of MMP is a direct reflection of the effect of GA on mitochondrial activity, which could enable the caspase family and lead to apoptosis in H_9_C_2_ cells. And antiapoptotic Bcl-2 and proapoptotic Bax proteins could regulate MMP. Bax levels were clearly elevated (*P* < 0.05) whereas Bcl-2 levels were significantly lowered (*P* < 0.05; Figures 4(b) and 4(c)) after GA exposure. These findings indicate that GA-induced cell injury could be linked to the mitochondrial apoptotic pathway.

### 3.3. GA Stimulated ROS by Regulating the Keap1-Nrf2 Signaling Pathway

Flow cytometry and DCFH-DA fluorescent testing were used to determine the ROS levels of H_9_C_2_ cells displaying green fluorescence. As we can see, the levels of ROS in the H_9_C_2_ cells rose in a dose-dependent way after GA treatment (*P* < 0.05; Figures 5(a) and 5(b)). These results confirm that GA causes the generation of ROS. And we investigated whether the generation of ROS was caused by a change in the Keap1-Nrf2 signaling pathway. In vitro RT-qPCR assessment of Keap1 and Nrf2 gene expression was performed, as presented in Figure 6(a). GA treatment upregulated Keap1 gene expression (*P* < 0.05) and downregulated Nrf2 gene expression in H_9_C_2_ cells. The activation of Nrf2 signaling was stimulated by a pressure-overload by GA over 24 h, which may be linked to the overproduction of ROS. Antioxidant defense is mostly regulated by Nrf2.

The article "Regulation of the Keap1-Nrf2 Signaling Axis by Glycyrrhetinic Acid Promoted Oxidative Stress-Induced H9C2 Cell Apoptosis" was published in 2022. Journal: Evid Based Complement Alternat Med.

GA treatment resulted in a marked increase in the Nrf2-dependent protein expression of HO-1. Western blotting revealed that GA administration increases Nrf2 and Keap1 protein expression in the cytoplasm and decreases Nrf2 protein expression inside the nucleus (*P* < 0.05; Figures 6(b) and 6(c)).

## 4. Discussion

The cardiotoxicity of drugs is a serious concern for clinical institutions, medical research institutes, and pharmaceutical companies. In this research, we used H_9_C_2_ cells to probe the mechanism of in vitro GA-induced heart damage. The present study found that GA-induced H_9_C_2_ cell apoptosis is dependent on excessive mitochondria-derived ROS. And GA also gives rise to a dynamic imbalance of oxidative and antioxidant systems. Furthermore, this apoptosis was based on the Keap1-Nrf2 signaling pathway.

H_9_C_2_ cells, a subclone of the primitive clonal cell line obtained from embryonic BD1X rat heart tissue, are commonly used to investigate cardiotoxicity in vitro [25]. To clarify the molecular mechanism of GA-induced cardiotoxicity in H_9_C_2_ cells, firstly we evaluated the cytotoxicity of GA. After H_9_C_2_ cells were fixed with 15–45 *μ*M GA, we found significant decreases in cell survival occurring in a concentration- and time-dependent way. Moreover, GA also significantly increased the leakage rate of LDH in the culture buffer (*P* < 0.05). The morphology of cardiomyocytes changed, and their numbers decreased. Thus, GA can induce cardiotoxicity *in vitro*.

Numerous studies have clarified that the production of intracellular ROS is closely related to apoptosis [26]. And mitochondria are a major generator of ROS, as the Nrf2 pathway is a biological sensor for chemically produced ROS [27]. In our study, GA induced the generation of ROS in cardiomyocytes in a dose-dependent manner (*P* < 0.05). The final accumulated ROS can initiate changes in the depolarization of the MMP. Our results indicated that GA administration increases the green fluorescence of cardiomyocytes, resulting in a drop in MMP and a reduction in the red/green fluorescence proportion, eventually leading to caspase-3 activation and cell apoptosis induction.

The article "Regulation of the Keap1-Nrf2 Signaling Axis by Glycyrrhetinic Acid Promoted Oxidative Stress-Induced H9C2 Cell Apoptosis" was published in 2022. Journal: Evid Based Complement Alternat Med.

Various stimulations, such as oxidative stress, could activate the mitochondrial apoptotic pathway [28]. Our research showed that mitochondrial malfunction occurs following GA exposure, which implies that mitochondria act as an important part of GA-induced apoptosis. This route involves the Bcl-2 family, which comprises numerous critical apoptosis-dependent proteins like the antiapoptotic protein Bcl-2 and the proapoptotic protein Bax. Furthermore, the ratio of Bax to Bcl-2 decides the transition of mitochondrial permeability [29]. The destruction of mitochondrial membrane permeability causes cytochrome C to be released, which binds to and oligomerizes Apaf-1. Then the oligomeric Apaf-1 mediates the cytochrome C-dependent activation of caspase-9, a lethal proteolytic enzyme that causes caspase-3 cleavage, PARP activation, and apoptosis [30]. The results of this experiment revealed that the expression of Bax in the GA dose groups was higher than that in the blank control group, whereas the expression of Bcl-2 protein in the former was lower than that in the latter. The level of Bax/Bcl-2 protein expression was dramatically raised (*P* < 0.05). Cleaved PARP/PARP, cleaved caspase-9/caspase-9, and cleaved caspase-3/caspase-3 protein expression levels all rose significantly following GA treatment.

The ROS makes a real difference in the activation of the caspase cascade produced by mitochondria, and the Nrf2 pathway is a major part of the cellular defense against oxidative stress [31]. Nrf2 dissociates from Keap1 on exposure to oxidative stress and then translocates into the nucleus, where it induces the expression of antioxidant genes, for example, HO-1. Previous research showed that the Nrf2 signaling pathway controls HO-1 expression [32]. GA dramatically lowered the expression levels of Nrf2 protein in the nucleus, Nrf2 target gene, and HO-1 protein levels but increased the levels of Keap1 and Nrf2 in the cytoplasm (*P* < 0.05). We thus conclude that the Keap1-Nrf2 signaling axis is implicated in GA-induced intracellular ROS generation and apoptosis.

## 5. Conclusion

In conclusion, the present findings indicated that GA significantly induced apoptosis of H_9_C_2_ cells. The underlying mechanism of cardiotoxicity of GA may not only involve the regulation of the Keap1-Nrf2 pathway but also the activation of mitochondrial-dependent caspase. Our work preliminarily explores the toxic effects and mechanisms of GA on myocardial cells and provides a basis for the safe application of GA.

The article "Regulation of the Keap1-Nrf2 Signaling Axis by Glycyrrhetinic Acid Promoted Oxidative Stress-Induced H9C2 Cell Apoptosis" was published in 2022. Journal: Evid Based Complement Alternat Med.

## Figures and Tables

**Figure 1:** Injurious effect of GA on H_9_C_2_ cells. (a) GA's Chemical structure. (b) Cell viability of H_9_C_2_ cells treated for 24 or 48 h with the indicated doses of GA and evaluated by CCK-8 assay. (c) Changes in the LDH release of H_9_C_2_ cells treated with GA. (d) Morphological alterations in H_9_C_2_ cells following GA treatment. Scale bar = 100 *μ*m. Values are expressed as the mean ± SD of three independent experiments. ^*∗*^*P* < 0.05 vs. the control group.

**Figure 2:** Effect of GA on the apoptosis of H_9_C_2_ cells. H_9_C_2_ cells were pretreated for 24 h with 15, 30, and 45 M GA. (a) H_9_C_2_ cells revealed GA-induced chromatin constriction after Hoechst 33242 and propidium iodide (PI) staining. Scale bar = 100 *μ*m. Apoptotic H_9_C_2_ cells were labeled with annexin V-FITC and PI for flow cytometry. (b) Raw flow cytometry data. (c) Apoptosis rates. Values reflect the mean ± SD of three independent experiments. ^*∗*^*P* < 0.05 vs. the control group.

**Figure 3:** Effect of GA on apoptosis-related proteins. H_9_C_2_ cells were pretreated for 24 h with 15, 30, and 45 M GA. (a, b) GA treatment increased cleaved PARP, cleaved caspase-3, and caspase-9 expression. ADR, adriamycin (positive control for the mitochondrial apoptosis test). Values reflect the mean ± SD of three independent experiments.^*∗*^*P* < 0.05 vs. the control group.

**Figure 4:** Effect of GA on the mitochondrial pathway of H_9_C_2_ cells. H_9_C_2_ cells were pretreated for 24 h with 15, 30, and 45 M GA. (a) JC-1 was used to stain H_9_C_2_ cells, and the MMP was examined using a fluorescent microscope. Scale bar: 100 *μ*m. (b, c) GA boosted Bax expression but decreased Bcl-2 expression. ADR, adriamycin (positive control for the mitochondrial apoptosis test). Values reflect the mean ± SD of three independent experiments.^*∗*^*P* < 0.05 vs. the control group.

**Figure 5:** Effects of GA on ROS. H_9_C_2_ cells were pretreated for 24 h with 15, 30, and 45 M GA. (a) Cellular ROS levels were measured by DCFH-DA flow cytometry after examination under a fluorescent microscope. Scale bar: 100 *μ*m. (b) ROS staining was studied quantitatively. H_2_O_2_ was used as a positive control. Values reflect the mean ± SD of three independent experiments.^*∗*^*P* < 0.05 vs. the control group.

**Figure 6:** Effects of GA on Keap1-Nrf2 signaling. H_9_C_2_ cells were pretreated for 24 h with 15, 30, and 45 M GA. (a) GA treatment increased the expression of the Keap1 gene but decreased that of the Nrf2 gene in H_9_C_2_ cells. (b, c) GA treatment increased the protein expression of HO-1, Nrf2, and Keap1 in the cytoplasm but decreased the protein expression of Nrf2 in the nucleus of H_9_C_2_ cells. H_2_O_2_ was used as a positive control. Values reflect the mean ± SD of three independent experiments.^*∗*^*P* < 0.05 vs. the control group.

The article "Regulation of the Keap1-Nrf2 Signaling Axis by Glycyrrhetinic Acid Promoted Oxidative Stress-Induced H9C2 Cell Apoptosis" was published in 2022. Journal: Evid Based Complement Alternat Med.

## Data Availability

All data generated or analyzed during this study are included within the article.

## Abbreviations

ROS: Reactive oxygen species
GA: Glycyrrhetinic acid
Nrf2: NF-E2-related factor 2
HO-1: Heme oxygenase-1
CCK-8: Cell Counting Kit-8
FITC: Fluorescein isothiocyanate
PI: Propidium iodide
OD: Optical density
ECL: Enhanced chemiluminescence
MMP: Mitochondrial membrane potential
NRVMs: Neonatal rat ventricular myocytes
DMEM: Dulbecco's modified Eagle's medium
PBS: Phosphate-buffered saline.

## Additional Points

ROS plays a key role in the activation of the caspase cascade induced by mitochondria. GA-induced cardiotoxicity is related to the overproduction of ROS. The Keap1-Nrf2 signaling axis is the most important endogenous antioxidant signaling axis. The Nrf2 pathway is a cellular sensor that induces ROS.
